RETRACTED

# 5-Aminolevulinic Acid-Based Photodynamic Therapy Pretreatment Mitigates Ultraviolet A-Induced Oxidative Photodamage

**DOI:** 10.1155/2018/9420745

**Published:** 2018-11-07

**Authors:** Hui Hua, Jiawei Cheng, Wenbo Bu, Juan Liu, Weiwei Ma, Chenchen Si, Jie Wang, Bingrong Zhou, Dan Luo

**Affiliations:** ^1^Department of Dermatology, The First Affiliated Hospital of Nanjing Medical University, Nanjing 210029, China; ^2^Institute of Dermatology, Chinese Academy of Medical Sciences (CAMS) & Peking Union Medical College (PUMC), Nanjing, Jiangsu, China

## Abstract

**Aim:**

To determine whether 5-aminolevulinic acid-based photodynamic therapy (ALA-PDT) is effective in combating ultraviolet A- (UVA-) induced oxidative photodamage of hairless mice skin *in vivo* and human epidermal keratinocytes *in vitro*.

**Methods:**

In *in vitro* experiments, the human keratinocyte cell line (HaCaT cells) was divided into two groups: the experimental group was treated with ALA-PDT and the control group was left untreated. Then, the experimental group and the control group of cells were exposed to 10 J/m^2^ of UVA radiation. ROS, O_2_^−^ species, and MMP were determined by fluorescence microscopy; p53, OGG1, and XPC were determined by Western blot analysis; apoptosis was determined by flow cytometry; and 8-oxo-dG was determined by immunofluorescence. Moreover, HaCaT cells were also treated with ALA-PDT. Then, SOD1 and SOD2 were examined by Western blot analysis. In *in vivo* experiments, the dorsal skin of hairless mice was treated with ALA-PDT or saline-PDT, and then, they were exposed to 20 J/m^2^ UVA light. The compound 8-oxo-dG was detected by immunofluorescence.

**Conclusion:**

In human epidermal keratinocytes and hairless mice skin, UVA-induced oxidative damage can be prevented effectively with ALA-PDT pretreatment.

## 1. Introduction

Skin photodamage has become a major public health issue given the tremendous increase in the number of patients suffering from it. Skin photodamage is caused by excessive exposure to ultraviolet (UV) radiation of the sun [1–4]. Ultraviolet radiation can cause acute reactions, such as erythema and edema; moreover, constant exposure to UV radiation can also lead to chronic skin reactions, such as photoaging and carcinoma [5, 6].

The major source of UV radiation is sunlight. There are two types of UV radiation that can reach the earth's atmosphere: UV radiation A (UVA) and UV radiation B (UVB), of which UVA constitutes 95%. Compared to UVB, the wavelength of UVA is longer; therefore, UVA penetrates deeper into the skin than UVB. Recent studies have reported that UVA is probably more mutagenic than UVB [7]. The UVA-induced skin damage may be indirect; it can trigger excessive production of ROS, which causes oxidative damage to proteins, lipids, and DNA. This leads to the generation of several types of oxidative products, such as 7,8-dihydro-8-oxo-guanosine (8-oxoG) and 8-oxo-7,8-dihydro-2′-deoxyguanosine (8-oxo-dG) [8, 9]. If the human body fails to remove UV mutagenic photoproducts within a definite period of time, the DNA cannot be repaired completely. These adverse products finally lead to the development of skin cancer.

RETRACTED

Skin photodamage can be prevented by adopting effective measures of UV protection. Currently, sunscreen lotions and protective clothing are the most effective photoprotective measures [10, 11]; however, many people find it difficult to use them on a regular basis. Previous studies have shown that these strategies have only caused a modest reduction in actinic keratosis (AKs) and squamous cell carcinomas (SCCs) of the skin; however, there has been no reduction in basal cell carcinomas (BCCs) of the skin [12, 13]. Some ingredients in sunscreens, such as benzophenone-3 (BP-3), can cause skin irritation and phototoxicity in susceptible populations; BP-3 is extensively used in organic sunscreens [14]. Currently, there is no worldwide consensus on the testing and labeling of sunscreens that offer UVA protection [15]. In fact, sunscreen alone may not be able to provide adequate protection from ultraviolet A. Therefore, it is very important to develop targeted chemoprevention strategies.

5-Aminolevulinic acid-based photodynamic therapy (ALA-PDT) is a noninvasive therapy; photosensitizer, oxygen, and light are the key components of ALA-PDT. Moreover, ALA is a precursor of protoporphyrin IX (PpIX). A topical formulation of ALA is used to target skin tissues; light of appropriate wavelength is used to activate the photosensitizer, which produces reactive oxygen species (ROS). Ultimately, this leads to cell necrosis and apoptosis [16, 17]. Previous studies have shown that ALA-PDT has a therapeutic effect on a variety of photodamage diseases, such as skin tumors and photoaging [18, 19]; moreover, it also prevents the onset of photodamage diseases, such as nonmelanoma skin cancers (NMSCs) and actinic keratoses (AKs). Goldberg et al. conducted a study on patients with a history of NMSCs and multiple AKs; they found that the onset of NMSCs can be prevented and delayed in these patients [20]. Togsverd-Bo et al. conducted a study on high-risk renal transplant recipients; they found that the onset of AK was significantly delayed when patients' normal skin was treated with repeated PDT for a long period of time [21]. The results indicate that ALA-PDT can prevent the occurrence of photodamage diseases, but we still do not know the exact mechanism through which ALA-PDT exerts inhibitory effect on UV-induced damages. In this study, hairless mice skin and HaCaT cells were pretreated with ALA-PDT. Then, they were exposed to UVA radiation to determine whether UVA-induced photodamage can be prevented with ALA-PDT pretreatment. We also determined the potential mechanisms through which ALA-PDT inhibits UVA-induced photodamage. The results indicate that UVA-induced DNA damage can be significantly reduced by ALA-PDT pretreatment, which upregulates p53-dependent DNA repair and activates the antioxidant enzymes. This indicates that UVA-induced oxidative damage can be inhibited with ALA-PDT pretreatment.

RETRACTED

## 2. Material and Methods

### 2.1. Cell Culture, ALA-PDT Treatment, and UVA Irradiation

The immortalized human keratinocyte cell line (HaCaT) was grown at 37°C in a humidified atmosphere of 5% CO_2_; the cell culture medium was Dulbecco's modified Eagle's medium (DMEM), which was supplemented with 10% fetal bovine serum (FBS) and 1% penicillin-streptomycin. Thereafter, HaCaT cells were subcultured by trypsinization, and they were used in subsequent passages. Under standard conditions, HaCaT cells were grown to >70% confluency. Then, subsequent experiments were performed. The cells were divided into three groups, namely, control group, UVA group, and ALA-PDT + UVA group. No treatment was provided to cells in the control group. In the UVA group, cells were irradiated with 10 J/cm^2^ of UVA light. In the ALA-PDT + UVA group, cells were incubated with 0.5 mmol/L of ALA for 4 h. Then, the cells were exposed to red laser light of 3 J/cm^2^ intensity (50 mW/cm^2^ for 60 s). Finally, these cells were irradiated with 10 J/cm^2^ of UVA light (3.7 mW/cm^2^ for 45 min). The UVA radiation was delivered using a UVA fluorescent lamp (340–400 nm wavelength, a peak at 305 nm, Sigma SS-04P, Shanghai, China). The intensity of UVA radiation was measured with a UV radiometer (Philips, Amsterdam, Netherlands). Before irradiating the cells with UVA light, the medium was removed and the cells were covered with a thin layer of phosphate-buffered saline (PBS).

### 2.2. Cell Viability Measurement

Cell viability was measured using a CCK-8 Kit (Beyotime Biotechnology, Shanghai, China). In brief, HaCaT cells (2000/100 *μ*L) were seeded into 96-well plates. Then, they were treated with ALA-PDT and UVA alone or in combinations. Thereafter, cells of each well were incubated with 10 *μ*L of CCK-8 solution for 2 h. To determine cell density, we measured the absorbance of cell culture at 450 nm with a Thermo Scientific Microplate Reader.

### 2.3. Measurement of Intracellular ROS and O_2_^−^

A fluorescent probe was used to measure the intracellular ROS and O_2_^−^ species produced by HaCaT cells. Cells were plated in 6-well plates or 96-well plates. Then, they were incubated in the dark with 10 *μ*mmol/L DCFH-DA or 5 *μ*mmol/L Dihydroethidium for 20 min at 37°C (Beyotime Biotechnology, Shanghai, China). The fluorescence intensity was measured with a SpectraMax 190 microplate reader (Molecular Devices, Sunnyvale, USA). Cells were observed under a fluorescence microscope, and they were also photographed randomly by a Nikon camera with constant time, exposure, and gain (Nikon, Tokyo, Japan).

RETRACTED

### 2.4. Flow Cytometry Analysis of Apoptosis

HaCaT cells had been treated with ALA-PDT by the abovementioned process. Then, these cells were harvested and washed with PBS. Finally, these cells were double-stained with an Annexin-V-FITC apoptosis detection kit (Beyotime Biotechnology, Shanghai, China). The cells were incubated with PI (10 *μ*L) and Annexin-V-FITC (5 *μ*L) at room temperature for 15 min in the dark. Then, they were quantitatively analyzed with a FACScan flow cytometer (BD, Franklin Lakes, NJ, USA). Cells stained with Annexin-V(+)/PI(−) were apoptotic in nature.

### 2.5. Evaluation of Mitochondrial Membrane Potential (MMP)

The fluorescent probe JC-1 (Beyotime Biotechnology, Shanghai, China) was used to determine the mitochondrial membrane potential (MMP) of HaCaT cells. Cells were cultured in 96-well plates and 6-well plates; these cells were incubated with JC-1 staining solution (5 *μ*g/mL) for 20 min at 37°C and rinsed twice with JC-1 staining buffer. A fluorescence microscope (Nikon, Tokyo, Japan) was used to determine the relative amounts of dual emissions from mitochondrial JC-1 monomers (490 nm excitation and 530 nm emission) or aggregates (525 nm excitation and 590 nm emission). The fluorescence intensity of mitochondrial JC-1 monomers and aggregates was determined with a SpectraMax 190 microplate reader (Molecular Devices, Sunnyvale, USA). An increase in the green/red fluorescence intensity ratio indicates mitochondrial depolarization.

### 2.6. Immunofluorescence Analysis for Detection of 8-Oxo-dG

HaCaT cells were cultured on coverslips and fixed in 4% paraformaldehyde for 15 min. Then, they were permeabilized with 0.5% Triton X-100 for 10 min. This blocked the nonspecific binding with PBS, which contained 1% bovine serum albumin (BSA) for 30 min. Then, they were incubated overnight with anti-8-oxo-dG monoclonal antibody at 4°C (1 : 800; Trevigen, Gaithersburg, USA). Subsequently, cells were washed again and incubated with Cy3-conjugated secondary antibody (1 : 1000, Beyotime Biotechnology, Shanghai, China) for 2 h. After washing stained cells with PBS, photomicrographs were taken with a fluorescence microscope (Nikon, Tokyo, Japan). The 8-oxo-dG-positive nuclei appeared red in color.

RETRACTED

### 2.7. Western Blotting for Detection of SOD1, SOD2, p53, XPC, and OGG1

After treating HaCaT cells with ALA-PDT mentioned above, Western blot analysis was performed on these cells. Cells were lysed in a RIPA buffer (Beyotime Biotechnology, Shanghai, China). Protein concentrations were quantified with a bicinchoninic acid protein assay kit (BCA, Beyotime Biotechnology, Shanghai, China). Then, equal amounts of 20 *μ*g protein/sample were separated with sodium dodecyl sulfate polyacrylamide gel electrophoresis (SDS-PAGE). After transferring the samples into PVDF membranes, the samples were allowed to react with specific primary antibodies: SOD1 (1 : 1000; CST, Boston, MA, USA), SOD2 (1 : 500; CST), p53 (1 : 1000; Sigma, St. Louis, MO, USA), XPC (1 : 1000; CST), and OGG1 (1 : 500; Sigma). Subsequently, the cells were incubated with HRP-conjugated anti-mouse or anti-rabbit IgG for 2 h. Protein expression levels were determined with an enhanced chemiluminescence (ECL) detection system. *β*-Actin was used as an internal control.

### 2.8. Animal

All animal experiments were performed after receiving approval from the Animal Use Committee of Nanjing Medical University in China. We included 28 female BALB/c athymic nude mice, 4–6 weeks old, and the weight of each mouse was between 19 and 22 g. We purchased these mice from Model Animal Research Center of Nanjing University in China. After acclimatizing the mice to experimental conditions, they were randomly divided to three groups (10 animals in each group): the control group (no treatment), the ALA-PDT + UVA group (10% ALA + 12 J/cm^2^ PDT + 20 J/cm^2^ UVA), and the UVA group (saline + 20 J/cm^2^ UVA).

### 2.9. ALA-PDT Treatment and UVA Irradiation

A piece of medical cotton was soaked with a specific concentration of ALA solution (10%; Fudan-Zhangjiang Bio-Pharmaceutical Co., Shanghai, China). Then, the cotton soaked with ALA solution was applied on approximately 4.0 cm^2^ of dorsal skin. In the UVA group, physiological saline was used as a negative control. The treated areas were covered with layers of plastic wrap and black plastic sheeting, and they were secured with a medical tape. We removed these dressings after 2 h. The treated tissues were irradiated for 10 min with a PDT laser (XD-635AB; Fudan-Zhangjiang Bio-Pharmaceutical Co., Shanghai, China) of wavelength 635 nm; the energy density of the PDT laser was 12 J/cm^2^ (50 m W/cm^2^ for 4 min). The mice were treated with ALA-PDT or physiological saline for two days. After these mice were anesthetized with 0.4% chloral hydrate (0.1 mL/10 g), they were irradiated with 20 J/cm^2^ of UVA light (3.7 mW/cm^2^ for 90 min).

RETRACTED

### 2.10. Immunofluorescence Analysis of 8-Oxo-dG

After fixing the specimens in 4% paraformaldehyde, they were embedded in a paraffin bath. After blocking endogenous proteins, sections were incubated overnight at 4°C with anti-8-oxo-dG monoclonal antibody (1 : 1000; Trevigen, Gaithersburg, USA). After washing the sections with PBS, they were incubated with Cy3-labeled secondary antibodies (1 : 2000; Beyotime Biotechnology, Shanghai, China) at 37°C for 1 h. Then, the slides were observed and pictures were captured under a fluorescence microscope.

### 2.11. Statistical Analysis

Statistical analysis was performed using the SPSS software for Windows, version 16.0 (SPSS, Chicago, IL, USA). Statistical analysis was carried out by one-way analysis of variance (ANOVA) and Student-Newman-Keuls (SNK-q) test. Data are expressed as the mean ± SD for each group. The values of ^∗^*p* < 0.05 were considered to be statistically significant, and they are indicated in the figures.

## 3. Results

### 3.1. Sublethal Dose of ALA-PDT Induced Intracellular ROS

We determined whether sublethal doses of ALA-PDT affected intracellular ROS levels. We incubated HaCaT cells with 0.5 mmol/L of ALA for 4 h. Cells were exposed to 3 J/cm^2^ intensity of red laser light. The results of the CCK-8 assay indicated that there was no significant difference between the cell viability of the ALA-PDT group and the control group (*p* > 0.05) (Figure 1(a)). The ROS levels were determined by the fluorescent probe DCFH-DA. The HaCaT cells were treated with sublethal doses of ALA-PDT. Compared to the control group, these cells showed stronger green fluorescence and increased fluorescence intensity (*p* < 0.05; Figure 1(c)).

### 3.2. Sublethal Dose of ALA-PDT Increased the Levels of SOD1 and SOD2 Proteins

The expression of SOD1 and SOD2 proteins was tested by Western blot analysis to evaluate the level of antioxidant enzymes in HaCaT cells treated with a sublethal dose of ALA-PDT. Compared to the control group, the levels of SOD1 protein increased by 117.56%, 151.15%, and 123.66% in HaCaT cells treated with ALA-PDT at 24 h, 36 h, and 48 h, respectively. The levels of SOD2 protein in the ALA-PDT group increased by 64.94%, 86.36%, and 58.44% at 24 h, 36 h, and 48 h, respectively, compared to those of the control group (*p* < 0.05; Figure 1(b)).

### 3.3. ALA-PDT Pretreatment Reduces UVA-Induced Oxidative Damage

After irradiating HaCaT cells with UVA light, we assessed the extent of oxidative damage by measuring the amount of ROS and O_2_^−^ species generated in this process. The number of ROS and O_2_^−^ species increased tremendously in HaCaT cells when they were irradiated with UVA light. However, the UVA-induced oxidative damage was reduced significantly when HaCaT cells were subjected to ALA-PDT pretreatment: the number of ROS and O_2_^−^ species declined tremendously in HaCaT cells subjected to ALA-PDT pretreatment, and the fluorescence intensities were reduced by 34.54% and 35.44%, respectively (*p* < 0.05 and *p* < 0.05, respectively; Figure 2).

RETRACTED

### 3.4. ALA-PDT Pretreatment Inhibits UVA-Irradiated Cytotoxicity

The cytotoxic effects of UVA and ALA-PDT were determined by performing the CCK-8 assay. The results indicated that cell viability decreased by 36.14% at 24 h after the samples were irradiated with UVA light. However, ALA-PDT pretreatment reduced by 15.07% UVA-induced cytotoxicity in those UVA-irradiated HaCaT cells (*p* < 0.05; Figure 3(a)).

### 3.5. ALA-PDT Pretreatment Suppressed UVA-Induced Apoptosis

In this study, HaCaT cells were doubly stained with Annexin-V/PI. Then, the apoptosis rate of these cells was determined by flow cytometry. Annexin-V(−)/PI(−) cells are live cells and Annexin-V(+)/PI(−) cells are early-stage apoptotic cells. Annexin-V(+)/PI(+) cells are late-stage apoptotic or necrotic cells. The apoptosis rate was expressed as a percentage of apoptotic cells in total cells. As shown in Figure 3(b), the early and late-stage apoptosis was significantly increased with UVA light. Compared to the UVA group, apoptosis significantly decreased by 31.60% in HaCaT cells subjected to ALA-PDT pretreatment (*p* < 0.05).

### 3.6. ALA-PDT Pretreatment Alleviates the UVA-Induced Mitochondrial Dysfunction

In order to determine the effect of ALA-PDT and UVA on mitochondria, we performed an assay to determine the changes in MMP by performing flow cytometry with the lipophilic fluorochrome JC-1. The accumulation of JC-1 in mitochondria led to the formation of JC-1 aggregates detected in the red channel. When the MMP was depolarized, JC-1 remained in the cytoplasm as monomers; these monomers were detected in the green channel. As shown in Figure 3(c), control cells exhibited bright red fluorescence. This indicated that control cells had a strong MMP. After being exposed to UVA, cells typically lost their MMP. Mitochondrial fluorescence intensity was undetected in these cells. The UVA-induced reduction of MMP can be significantly prevented by subjecting HaCaT cells to ALA-PDT pretreatment.

### 3.7. ALA-PDT Pretreatment Inhibited the Level of 8-Oxo-dG

Immunofluorescence detected 8-oxo-dG, which is the characteristic product of UVA-induced oxidative damage on DNA. When HaCaT cells were exposed to UVA, there was a significant increase in 8-oxo-dG generation. However, ALA-PDT pretreatment could significantly reduce the elevated levels of 8-oxo-dG in HaCaT cells subjected to UVA light (*p* < 0.05; Figure 4(a)). *In vivo*, we also observed that UVA light induced the production of 8-oxo-dG in the skin of hairless mice; however, ALA-PDT can inhibit the excessive generation of 8-oxo-dG in the skin of hairless mice, which was exposed to UVA radiation (*p* < 0.05; Figure 4(b)).

RETRACTED

### 3.8. ALA-PDT Pretreatment Increased the Levels of p53, XPC, and OGG1 Proteins

To determine whether ALA-PDT pretreatment can increase the expression level of proteins involved in DNA damage repair, we determined the expression of p53, XPC, and OGG1 proteins in HaCaT cells by Western blot analysis. The results indicated that compared to the unirradiated group, the expression of p53, XPC, and OGG1 proteins significantly increased by 36.48%, 48.97%, and 136.45% in the UVA-irradiated group (*p* < 0.05). In the ALA-PDT pretreatment group, the levels of p53, XPC, and OGG1 significantly increased by 25.38%, 33.80%, and 29.64%, respectively, than those in the UVA group (*p* < 0.05; Figure 5).

## 4. Discussion

When human epidermal keratinocytes and the skin of hairless mice were pretreated with ALA-PDT, the UVA-induced oxidative damage was reduced significantly. ROS plays a significant role in the mechanism of ALA-PDT [22]. High-level ROS can disrupt cellular processes, while low-level ROS can mediate cellular signaling [23]. Moreover, ROS can elicit oxidative damage and apoptosis in photoaged fibroblasts, which may be the basis for the rejuvenating effects on photoaged skin [24]. The mechanism of acne treatment is as follows: ROS suppresses the expression of IL-1*α* on keratinocyte hyperkeratosis via the FGFR2b pathway [25]. In our previous study, low concentration of ALA (0.5 mmol/L) and low intensity of red light (3 J/cm^2^) did not have a significant effect on cell viability; however, the p53-dependent pathway was activated sufficiently with excessive production of ROS. Therefore, a sublethal dose of ALA-PDT was used in subsequent cell experiments.

When HaCaT cells were exposed to UVA radiation, the production of reactive oxygen species (ROS) increased tremendously; the UVA radiation interacted with endogenous chromophores to produce ROS, such as superoxide radical (O_2_^−^) and singlet oxygen (O_2_). The reactive oxygen species can cause damage to cellular proteins, lipids, and DNA, which leads to the formation of oxidative DNA lesions [26]. Moreover, 8-oxo-dG is a characteristic biomarker of DNA oxidation because guanine bases are most susceptible to oxidation [27]. Hu et al. pretreated keratinocytes with oxyresveratrol or kuwanon O; the two phenolic compounds were extracted from the roots of *Morus australis*. They reported both of them were able to inhibit the generation of ROS in keratinocytes, which were irradiated with UVA, and enhanced the cell viability and antioxidative defense capability of keratinocytes [28]. In our study, when HaCaT cells were exposed to UVA light, it increased the generation of ROS, O_2_^−^, and 8-oxo-dG species. Moreover, ALA-PDT pretreatment protected HaCaT cells from UVA-induced damage by suppressing the generation of cellular ROS, O_2_^−^, and 8-oxo-dG.

RETRACTED

UVA-mediated apoptosis was partially induced indirectly by generating ROS. It has been well established that after being exposed to UVA light, keratinocytes undergo apoptosis [29–31]. When HaCaT cells were exposed to UVA, apoptosis was induced in these cells; the signs of apoptosis were as follows: cell viability decreased, the fragmentation of DNA increased, and cell morphology is alerted. A previous study reported that ellagic acid pretreatment can successfully suppress UVA-induced apoptosis [32]. In our study, we proved that ALA-PDT pretreatment could successfully suppress UVA-induced apoptosis in HaCaT cells. Complex pathways are involved in the initiation and progression of UV-mediated apoptosis of keratinocytes. Mitochondrial-, death receptor-, ER stress-, and ROS-mediated apoptosis have been reported in these studies [33, 34]. Petruk et al. reported that *Opuntia* raw extract, which is a phenolic antioxidant, was able to protect cells against UVA-induced apoptosis by inhibiting the activation of caspase-3 and caspase-7 [35]. We confirmed that MMP of HaCaT cells was significantly affected by UVA radiation; moreover, ALA-PDT pretreatment can significantly protect HaCaT cells against UVA-induced mitochondrial damage. This observation completely complies with a previous report, which states that ellagic acid protects keratinocytes against UVA-induced apoptosis through the mitochondrial apoptotic pathway [32].

Skin diseases are caused by UVA-induced oxidative damage and apoptosis [36–38]. In order to effectively prevent UVA-induced photodamage, endogenous antioxidants must be induced and DNA repair capacity must be improved [39]. Several studies have reported that T-oligos induced a protective DNA-damage response by activating p53, leading to the upregulation of antioxidant enzymes and DNA-repair enzymes. This protects the DNA from future insults [40–42]. The inducible DNA damage response, which is also known as SOS response, was first found in bacteria. Adaptive DNA damage responses are elicited in cells by administering sublethal doses of DNA-damaging agents [43, 44]. And a transient increase in DNA repair rate was observed by following acute sublethal DNA damage [45].

RETRACTED

Reactive oxygen species (ROS)/free radicals were scavenged from a network of antioxidant enzymes, thereby maintaining cellular redox homeostasis [36, 46]. Superoxide dismutases (SODs), especially copper and zinc-dependent superoxide dismutase (SOD1) and the mitochondrial manganese-dependent superoxide dismutase (SOD2), efficiently catalyze the conversion of super oxides into oxygen and hydrogen peroxides. It is well known to be a major antioxidant enzyme that protects cells from oxidative stress, and it prevents carcinogenesis [47–49]. Effect of UVA irradiation on antioxidant enzymes has been reported. Skin cells prepare for subsequent exposure to damaging radiation by upregulating the activities of the antioxidant enzymes SOD1 and SOD2, which also demonstrated the existence of an SOS-like adaptive response [50]. Lee et al. reported that T-oligo can induce antioxidant defenses by upregulating the expression of SOD1 and SOD2 [40]. It is also reported that when chronically irradiated mouse skin was topically treated with T-oligo, the level of 8-oxo-dG reduced substantially [51]. Our data was completely compliant with the above observation: the expression of SOD1 and SOD2 was induced and activated with sublethal doses of ALA-PDT, which offered protection against oxidative stress. We speculate that ALA-PDT protects cells from UVA-induced damage by reducing the generation of ROS and 8-oxo-dG. Thus, apoptosis of cells is suppressed by ALA-PDT, which mainly induces antioxidant defenses. SODs are important antioxidant components of antioxidant systems. However, the activation mechanisms of SODs are still unclear. It has been reported that bread crust extract could activate SOD through the receptor for advanced glycation end products (AGEs). But high doses of bread crust extract are independent of AGE receptors, indicating that additional mechanisms are involved in the activation of SOD [52]. In our experiments, sublethal doses of ALA-PDT induced an antioxidant response by activation of SOD1 and SOD2, but the specific activation mechanism of SODs remained to be further studied.

The main objectives of DNA repair mechanisms are as follows: (i) to ensure genomic stability and (ii) to eliminate DNA lesions [53, 54]. The ubiquitous DNA oxidation product 8-oxo-dG is repaired predominantly via base excision repair (BER) pathway and nucleotide excision repair (NER) pathway [55]. The BER DNA glycosylase 8-oxoguanine DNA glycosylase 1 (OGG1) dominates the repair of 8-oxo-dG; the minor contributor is xeroderma pigmentosum group C (XPC), which is related to nucleotide excision repair (NER) [26, 56, 57]. The tumor suppressor p53 is closely related to the NER pathway, which promotes the expression of XPC protein and improves NER [58]. Previous studies have reported that p53 coordinates the BER pathway to prevent genomic instability [59]. In our study, the levels of OGG1 and XPC proteins can be improved with ALA-PDT pretreatment. The above results indicate that ALA-PDT can induce NER- and BER-based DNA damage repair by activating p53, which accelerates the removal of 8-oxo-dG and reduces apoptosis.

RETRACTED

A hairless mouse skin model was used to determine whether the protective DNA damage response was elicited *in vivo*. The *in vivo* results indicate that the expression of 8-oxo-dG was significantly reduced with ALA-PDT pretreatment. However, we failed to observe sunburn cells and TUNEL-positive cells in hairless mice skin. This observation completely complied with previous reports, stating that sunburn cells are absent or rare *in vivo* after being exposed to UVA; however, UVA can induce apoptosis in cultured cells [60, 61].

In summary, our results prove that ALA-PDT pretreatment can exert antioxidative damage by reducing the generation of ROS, O_2_^−^, and 8-oxo-dG, as well as diminishing the apoptosis of cells. We also elucidated the possible molecular mechanisms through which sublethal doses of ALA-PDT induced protective DNA damage responses in human keratinocytes. The inducible antioxidant responses are as follows: the p53-dependent upregulation of DNA repair capacity and the activation of antioxidant enzymes. These antioxidant responses can protect skin cells from oxidative photodamage, which is induced by UVA light. Thus, ALA-PDT might be used for the prevention of diseases due to oxidative damage. However, in addition to the inducible antioxidant responses, more detailed studies on their antioxidant mechanism are still needed. Wang and Sun have reported that ALA-PDT suppressed IFN-*γ*-induced K17 expression in HaCaT cells via the MAPK pathway [62]. The MAPK signaling pathway is involved in many biological processes, such as cell proliferation, differentiation, gene expression, and apoptosis [63]. Further experiments are required to determine whether the MAPK pathway participated in the process of ALA-PDT exerting antioxidant effects. Also, our present experiments have failed to fully confirm whether ALA-PDT can prevent UVA-induced photodamage *in vivo*. In subsequent studies, we will further confirm whether ALA-PDT exerts photoprotective effect by eliciting an SOS-like response *in vivo*. The possibility of using ALA-PDT for skin photoprotection or the prevention of oxidative damage in humans deserves further investigation.

RETRACTED

## Figures and Tables

**Figure 1:** Sublethal doses of ALA-PDT induced intracellular ROS, and the expression levels of SOD1 and SOD2 were determined in HaCaT cells. The ALA-PDT group was treated with the following components: 0.5 mmol/L of ALA and 3 J/cm^2^ of red laser light. (a) Cell viability was detected by the CCK-8 assay at 450 nm after being treated with a sublethal dose of ALA-PDT. (b) The expression levels of SOD1 and SOD2 proteins were determined 24 h, 36 h, and 48 h after receiving a sublethal dose of ALA-PDT. Protein expression levels were quantified by using *β*-actin as a control. (c) Cells in the ALA-PDT group were treated with a sublethal dose of ALA-PDT. The intracellular ROS showed green fluorescence under a fluorescence microscope, and the fluorescence intensity was determined by a fluorescence microplate reader. Data were expressed as mean ± SD, *n* = 3 for each group, ^∗^*p* < 0.05, ^#^*p* > 0.05.

**Figure 2:** UVA-induced oxidative damage was reduced with ALA-PDT pretreatment. (a, b) Cells were treated with a sublethal dose of ALA-PDT, then these cells were irradiated with 10 J/cm^2^ of UVA light. Cells were incubated with 10 *μ*mmol/L DCFH-DA or 5 *μ*mmol/L Dihydroethidium for 20 min, after which ROS and O_2_^−^ production was visualized by fluorescence microscopy. Intracellular ROS and O_2_^−^ species exhibited green and red fluorescence under a fluorescence microscope; the fluorescence intensity was determined by a fluorescence microplate reader. Data were expressed as mean ± SD, *n* = 3 for each group, ^∗^*p* < 0.05.

**Figure 3:** ALA-PDT pretreatment inhibits cytotoxicity and apoptosis of cells irradiated with UVA. Cells were treated with a sublethal dose of ALA-PDT, then these cells were irradiated with 10 J/cm^2^ of UVA light. (a) The cell viability was detected by CCK-8 assay at 450 nm. (b) The apoptosis of HaCaT cells was measured by using Annexin-V and PI in conjunction with flow cytometry; Annexin-V(+)/PI(−) cells were early-stage apoptotic cells. (c) Early apoptosis was indicated by a decrease in mitochondrial membrane potential. When the fluorescence probe JC-1 underwent a transition from red light to green light, it indicated a decrease in cell membrane potential. This was an indicator of early apoptosis. The fluorescence intensity of the green/red ratio was determined by a fluorescence microplate reader. Data were expressed as mean ± SD, *n* = 3 for each group, ^∗^*p* < 0.05, ^#^*p* > 0.05.

**Figure 4:** The expression level of 8-oxo-dG was inhibited with ALA-PDT pretreatment. Cells were treated with a sublethal dose of ALA-PDT, then these cells were irradiated with 10 J/cm^2^ of UVA light. The expression level of 8-oxo-dG was detected by immunofluorescence. (a, b) Red fluorescence represented 8-oxo-dG-positive cells. Photographs were taken randomly under a fluorescence microscope, and the number of positive cells was counted; this represented the data for each group. Data were expressed as mean ± SD, *n* = 3 for each group, ^∗^*p* < 0.05.

RETRACTED

**Figure 5:** ALA-PDT pretreatment increased the levels of p53, XPC, and OGG1 proteins. Cells were treated with a sublethal dose of ALA-PDT, then these cells were irradiated with 10 J/cm^2^ of UVA light. A Western blot analysis was carried out to detect the expression levels of p53, XPC, and OGG1 proteins. Protein expression levels were quantified by using *β*-actin as control. Data were expressed as mean ± SD, *n* = 3 for each group, ^∗^*p* < 0.05.

## Data Availability

The data used to support the findings of this study are available from the corresponding author upon request.
